The article "Deep multi-modal intermediate fusion of clinical record and time series data in mortality prediction" was retracted in 2025. Reasons: plagiarism; overlap with other authors' work; concerns about the article.

# Deep multi-modal intermediate fusion of clinical record and time series data in mortality prediction

**DOI:** 10.3389/fmolb.2023.1136071

**Published:** 2023-03-08

**Authors:** Ke Niu, Ke Zhang, Xueping Peng, Yijie Pan, Naian Xiao

**Affiliations:** ^1^ Computer School, Beijing Information Science and Technology University, Beijing, China; ^2^ Australian Artificial Intelligence Institute, Faculty of Engineering and Information Technology, University of Technology Sydney, Sydney, NSW, Australia; ^3^ Department of Computer Science and Technology, Tsinghua University, Beijing, China; ^4^ EIT Institute for Advanced Study, Ningbo, China; ^5^ Department of Neurology, The Third Hospital of Xiamen, Xiamen, China; ^6^ Department of Neurology and Geriatrics, Fujian Institute of Geriatrics, Fujian Medical University Union Hospital, Fuzhou, China

**Keywords:** mortality prediction, time series, clinical records, multimodal fusion, contextual information

## Abstract

In intensive care units (ICUs), mortality prediction is performed by combining information from these two sources of ICU patients by monitoring patient health. Respectively, time series data generated from each patient admission to the ICU and clinical records consisting of physician diagnostic summaries. However, existing mortality prediction studies mainly cascade the multimodal features of time series data and clinical records for prediction, ignoring thecross-modal correlation between the underlying features in different modal data. To address theseissues, we propose a multimodal fusion model for mortality prediction that jointly models patients’ time-series data as well as clinical records. We apply a fine-tuned Bert model (Bio-Bert) to the patient’s clinical record to generate a holistic embedding of the text part, which is then combined with the output of an LSTM model encoding the patient’s time-series data to extract valid features. The global contextual information of each modal data is extracted using the improved fusion module to capture the correlation between different modal data. Furthermore, the improved fusion module can be easily added to the fusion features of any unimodal network and utilize existing pre-trained unimodal model weights. We use a real dataset containing 18904 ICU patients to train and evaluate our model, and the research results show that the representations obtained by themodel can achieve better prediction accuracy compared to the baseline.

## 1 Introduction

With the advancement of medical technology, patients in the Intensive Care Unit (ICU) are monitored by different instruments at the bedside that measure different vital signals Sun et al. (2021) about the patient’s health. Such as heart rate, systolic blood pressure, temperature, *etc.* This type of data is called time series data. Time series data has two characteristics of irregularity under the aspects of intra-series and inter-series. Intra-series irregularity is the irregular time intervals between observations within a time series. Inter-series irregularity is the different sampling rates among time series. During their stay, doctors visit the patient intermittently for check-ups and make clinical record about the patient’s health and physiological progress. These notes can be perceived as summarized expert knowledge about the patient’s state. This type of data is called clinical record data. Researchers based on these data can be used to make mortality predictions for patients, which facilitates hospitals to allocate medical resources appropriately and provide cost-effective resource services to patients who need them most. However, the above data have their own unique characteristics Niu et al. (2022b), such as temporality, high dimensionality, and heterogeneity, so it is a challenge to extract key features from the large amount of patient data for prediction tasks.

The article "Deep multi-modal intermediate fusion of clinical record and time series data in mortality prediction" was retracted in 2025. Reasons: plagiarism; overlap with other authors' work; concerns about the article.

In recent years, deep learning techniques have been widely used in the medical field, enabling the task of extracting key features of patients to achieve predictive modeling. In particular, Recurrent Neural Networks (RNN) and its variants Long Short Term Memory (LSTM) Hochreiter and Schmidhuber (1997) and Gated recurrent Unit (GRU) Cho et al. (2014) have been used to process time series data. Lipton et al. (2015) used LSTM to model patient clinical data to classify 128 diagnoses. Che et al. (2018) used GRU-d Pei et al. (2021) (GRU-based recurrent neural network) to model patient time series data generated from ICU to analyze missing values in the time series. Convolutional neural networks (CNN) and BERT models have also been widely used in medical prediction tasks. Grnarova et al. (2016) used convolutional neural networks (CNN) to construct document representations for mortality prediction tasks. Lee et al. (2020) proposed the BioBert model for use in various biomedical text mining tasks. However, most previous work used a single data source for mortality prediction without aggregating information from multiple sources of data, making the representation learned by the model incomplete.

Most previous work has used time series data for mortality prediction tasks. For example, Zhu et al. (2018) combined a bidirectional LSTM model with supervised learning to capture temporal changes in time series data and used the extracted time series features for ICU mortality prediction. Some researchers have also attempted to use clinical records for mortality prediction tasks. For example, Darabi et al. (2020) used transformer networks and the recently proposed BERT language model to embed these clinical record data streams into a unified vector representation for downstream mortality prediction tasks. However, in a real-world clinical setting, time series data can be missing due to different collection frequencies Sun et al. (2020), and thus time series data may be incomplete. On the other hand, clinical records may suffer from spelling errors, non-standard abbreviations, and different writing styles Qiao et al. (2019), making it difficult to use clinical annotations for prediction.

The article "Deep multi-modal intermediate fusion of clinical record and time series data in mortality prediction" was retracted in 2025. Reasons: plagiarism; overlap with other authors' work; concerns about the article.

To address the above issues, time series data and clinical records can be combined for mortality prediction, and these prediction tasks can benefit from complementary relationships in multimodal data Su et al. (2020). Huang et al. (2021) demonstrated mathematically that the quality of the latent representation space directly determines the effectiveness of multimodal learning models. And with sufficient training data, the richer the variety of modalities, the more accurate the estimation of the representation space and thus the better the multimodal learning model. Recently, several researchers have modeled both kinds of data for mortality prediction. For example, Yang et al. (2021) proposed a multimodal deep neural network that considers both time series data and more clinical records. In addition, chronic and non-chronic patients are classified when dealing with clinical records. Khadanga et al. (2019) proposed a multimodal neural network model that extracts features from both time series data and clinical records and derives multimodal features. For better processing of textual data information, Deznabi et al. (2021) proposed a fine-tuned Bert model to process textual data. Experiments showed that the model combining the two could improve the prediction accuracy compared to using only time series data or only clinical records.

However, existing multimodal models still have some limitations. Most models utilize different deep neural networks to model the modal data and then output feature representations of the modal data by connecting each modal feature representation Song et al. (2019) at the feature level, which is then used to predict the final outcome. Since different modal data usually have different properties, resulting in inconsistent spatial and temporal dimensions, this poses an obstacle to capturing potential interrelationships in the low-level feature space. The inclusion of the fusion module after extracting the data features also increases the complexity Yu et al. (2019) of the network and makes training more difficult.

The article "Deep multi-modal intermediate fusion of clinical record and time series data in mortality prediction" was retracted in 2025. Reasons: plagiarism; overlap with other authors' work; concerns about the article.

To address the above issues and challenges, we propose a multimodal fusion neural network model that combines time-series data as well as textual information from clinical annotations for predicting mortality. This task is defined as predicting whether a patient will die before discharge from the hospital based on data from the first 2 days. Our model uses a fine-tuned Bert model Devlin et al. (2018) to process the text part and generate textual feature vectors, and feeds the time series data into a Long Short Term Memory (LSTM) network and generates time series feature vectors. We improve a lightweight fusion module Su et al. (2020) by allowing the feature vectors of two equal feature blocks to enter the fusion module before cascading the prediction, thus capturing the correlation and important feature information between the underlying modal data. Correlations and important feature information between features, and finally, the obtained multimodal features are modeled through the GRU layer to capture the dependencies of multimodal features.

To sum up, the main contributions of this paper are as follows:

1) We introduce a fusion module to fuse multimodal features to improve the performance of the model. It can capture individual modal contextual information as well as the underlying feature correlation between different modalities.
2) We propose an end-to-end model, to accurately predict patient mortality risk based on multimodal fusion features in time series data and clinical records.
3) We conducted experiments on the mortality prediction task using a real dataset and showed that the proposed model outperformed all comparative methods.

The rest of this paper is organized as follows: Section 2 reviews the related work. Section 3 then presents the details of our model. In Section 4, we present the results of experiments performed on real datasets. Finally, we conclude our work in Section 5.

## 2 Related works

There are three main areas of related work: time series data mining and clinical record mining and multimodal learning, and we briefly discuss the latest work in this area.

### 2.1 Clinical time series data mining

In the area of mortality prediction for critically ill patients, most of the previous work has focused on using time series data of patients for prediction. Due to the long-term dependency problem among time series data, the most advanced results have been achieved since the PhysioNet Challenge Silva et al. (2012) in 2012 for long short term memory (LSTM) networks to process medical data. Harutyunyan et al. (2019) provided a preprocessing standard for the MIMIC III Johnson et al. (2016) database using LSTM models to handle in-hospital mortality prediction, loss of compensation prediction, length of stay prediction and phenotypic typing for four tasks. In this paper, recurrent neural networks are used for prediction. Other models also use different forms of recurrent neural networks to predict mortality outcomes. Liu and Chen (2019) proposed a novel selective recurrent neural network with randomly connected gating units (SRCGUs), which not only reduces the number of parameters and saves time, but also dynamically adjusts their importance weights Niu et al. (2022a) to select a more appropriate neural network for prediction.

The article "Deep multi-modal intermediate fusion of clinical record and time series data in mortality prediction" was retracted in 2025. Reasons: plagiarism; overlap with other authors' work; concerns about the article.

### 2.2 Natural language processing in medical text

For clinical records, researchers have attempted to apply natural language processing (NLP) to medical prediction tasks. Grnarova et al. (2016) proposed a convolutional document embedding method based on the unstructured textual content of clinical records and evaluated the mortality prediction task against the clinical records of MIMIC III. The open set of biomedical word vectors/embeddings proposed by Zhang et al. (2019) (BioWordVec) that integrates biomedical domain knowledge to better capture the semantics of specialized terms and concepts, and also improves the quality of word embeddings Zhang et al. (2020). However, one drawback of word embedding is that it cannot address multiple meanings because each word is represented by only one vector. Peters et al. (2018) proposed a context-based pre-training model (ELMO) that dynamically adjusts word embedding according to the context, which can address the problem of multiple meanings Liu et al. (2019) of a word. However, this model uses LSTM to extract features instead of Transformer, and many studies have demonstrated that Transformer is far more capable of extracting features than LSTM.

Recently, BERT-based models have been used in the medical field due to their phenomenal success in natural language processing (NLP). Many studies are based on BERT models for clinical applications. Darabi et al. (2020) trained BERT models on clinical records and produced results with timestamps. The obtained patient embeddings verified the validity of unstructured text data. Lee et al. (2020) investigated how the recently introduced pre-trained language model BERT can be applied to biomedical corpora and proposed a pre-trained biomedical language representation model (BioBERT) for biomedical text mining. The analysis results show that the pre-training of biomedical corpus helps BERT to understand complex biomedical texts.

### 2.3 Multi-modal learning

All these models use only one data source when making mortality predictions. However, Khadanga et al. (2019) showed that the combination of time series and clinical record is useful for ICU mortality prediction. They used a convolutional neural network (CNN) on top of the pre-trained word embedding Zhang et al. (2019) of to obtain a representation of clinical record and a long short term memory network (LSTM) to embed the time-series portion of the data. The two representations were then connected for prediction. Deznabi et al. (2021) also showed the usefulness of combining time series data with clinical record information. They used the LSTM model for the time series portion of the data and a fine-tuned BioBERT Lee et al. (2020) for the clinical record. The multimodal segmentation attention module proposed by Su et al. (2020) is able to fuse blocks of features in each channel direction and capture correlations Ilievski and Feng (2017) between feature vectors. The fusion module is designed to be compatible with features of various spatial dimensions and sequence lengths for both cnn and rnn. thus, the fusion module can be easily added to the fusion features of any unimodal network and utilize existing pre-trained unimodal model weights. Therefore, We will use a representation of the clinical record in conjunction with the time series portion of the patient data and incorporate the fusion module to improve the performance of in-hospital mortality prediction. In the next section, we will define the notation and method architecture.

The article "Deep multi-modal intermediate fusion of clinical record and time series data in mortality prediction" was retracted in 2025. Reasons: plagiarism; overlap with other authors' work; concerns about the article.

## 3 Methods

In this section, we first define some notations to describe both data and mortality prediction tasks. Then we will describe in detail the composition of the model, which consists of three parts: unimodal feature modeling, multimodal feature fusion, and mortality prediction module. Figure 1 shows an overview of the model.

**FIGURE 1:** The overall architecture of the model.

### 3.1 Notations

Each patient has a number of clinical records during his hospitalization, and the data are in the format of time t corresponding to one clinical record. For a patient p with k clinical records, we denote C(p) = Ct_1_, Ct_2_, …, Ct_*k*_, We also have time-series data collected during the patient’s stay as X(p) = X_1_, X_2_, X_3_, …, X_*t*_.

### 3.2 The overview of model

As shown in Figure 1, the model consists of a unimodal feature modeling module, a fusion module, and a mortality prediction module. We model the clinical records using a BERT-based fine-tuning model, and then feed each clinical record of the patient into the textual part of our model separately, and then combine the resulting embeddings to obtain a final representation of the textual part of the data. We use a Long Short Term Memory (LSTM) network to model the pre-processed time series data and generate time series embeddings Shi et al. (2021). We then propose an improved fusion module for fusing features of single modalities, which partitions each modality into equal blocks of features on a channel and creates a joint representation for generating soft attention across feature blocks for each channel. The correlation information and important feature information between different modal data is captured through the attention mechanism. The unimodal features are passed through the fusion module to generate a multimodal feature matrix. Finally, the multimodal feature representation is modeled through the GRU layer to capture the dependencies between multimodal features. To more comprehensively represent the medical information of patients, we combine the modeled multimodal feature representation with the time series representation for prediction.

The article "Deep multi-modal intermediate fusion of clinical record and time series data in mortality prediction" was retracted in 2025. Reasons: plagiarism; overlap with other authors' work; concerns about the article.

### 3.3 Single-modal feature modeling

The multimodal feature fusion module integrates different types of inputs. The feature extraction module of model includes time series data feature extraction and clinical record feature extraction.

#### 3.3.1 Time-series feature modeling

For the time series part of the model, our preprocessing followed the work of Harutyunyan and Khadanga et al. We limited the collection of time series data to 48 h after admission, for which we used untimed sampling. If a variable had a missing value Tan et al. (2019) at the collection node, we used the preset value of the feature given by Harutyunyan et al. (2019) After preprocessing the time series data, we used the LSTM network. We input the whole time series data of the patient into the LSTM model. LSTM is an RNN for capturing long-term dependencies Yoon et al. (2018) in serial data. It takes a sequence of {x_*t*_}^*T*^ of length T as input and outputs a sequence of {h_*t*_}^*T*^ say hidden state vectors of length T using the following equation.

$$i_{t}=\sigma \left(x_{t}W^{\left(xi\right)}+h_{t-1}W^{\left(hi\right)}\right)$$ (1)

$$f_{t}=\sigma \left(x_{t}W^{\left(xf\right)}+h_{t-1}W^{\left(hf\right)}\right)$$ (2)

$$c_{t}=f_{t}⊙c_{t-1}+i_{t}⊙tanh\left(x_{t}W^{\left(xc\right)}+h_{t-1}W^{\left(hc\right)}+b^{\left(c\right)}\right)$$ (3)

$$o_{t}=\sigma \left(x_{t}W^{\left(xo\right)}+h_{t-1}W^{\left(ho\right)}+b^{\left(o\right)}\right)$$ (4)

$$h_{t}=o_{t}⊙\sigma_{h}\left(c_{t}\right)$$ (5)

In each step, the LSTM combines the current input x_*t*_ with the previous hidden state h_*t*−1_ to generate the current hidden state h_*t*_; h_*t*_ = LSTM(x_*t*_, h_*t*−1_) for t = 1 to t = T.

#### 3.3.2 Clinical record feature modeling

Modeling clinical records requires capturing the interactions between different words Huang et al. (2021), and the Word2vec Church (2017) approach was previously used to model text, which is no longer considered the most effective approach with the advent of BERT. Bert-based models started to be used to capture word interactions, and these models also outperformed traditional NLP models in the field of text modeling. So we use Bert-based models to fine-tune the clinical records to obtain embeddings Peng et al. (2019) of each clinical record of a patient. Specifically, we used the BioBert model proposed by Alsentzer et al. (2019) for the text part, which fine-tunes the clinical records in the MIMIC III dataset.

The article "Deep multi-modal intermediate fusion of clinical record and time series data in mortality prediction" was retracted in 2025. Reasons: plagiarism; overlap with other authors' work; concerns about the article.

After initializing the text model to BioBert, we used the original BERT’s sentence classifier, which uses a classification token (CLS) to classify relationships. We added a softmax layer to the output of the classification token (CLS) for each clinical record separately and further adjusted the parameters of the model to predict the in-hospital mortality rate of the patients. Finally, we took the average embedding value of all clinical records of the patient to obtain the overall textual embedding value of the patient. This is shown in Eq. 6.

$$H_{C}=\frac{1}{N}\overset{N}{\underset{i=1}{\sum }}BCB\left(c_{t_{i}}\right)$$ (6)

### 3.4 Multi-modal feature fusion

In this section, we will detail the key part of the model, the multimodal feature fusion module. The flow chart of the algorithm is shown in Algorithm 1.

First, the time series and clinical record representations obtained in the modeling module are transformed into the same dimensions, and then their feature representations are input to the intermediate fusion module. The feature matrix of a single modality is divided into equal channel feature blocks. The number of channels in each block is C. We denote the set of feature blocks of time series modality t as R_*t*_, and we denote the set of feature blocks of clinical record modality c as R_*c*_. That is, R_*c*_ = (R_*c*1_, R_*c*2_, …, R_*cn*_) and R_*t*_ = (R_*t*1_, R_*t*2_, …, R_*tn*_), and n is the number of characteristic blocks.

The intermediate fusion module performs a concatenation operation on the modal features of each channel block to learn the global contextual information inside each modality. Taking the modal feature R_*c*_ as an example, we perform a summation operation on the modal feature R_*c*_ level to generate a shared representation H_*c*_, and then perform global average pooling in spatial dimension:

$$H_{c}=\underset{\left(R_{c1},R_{c2}...,,R_{cn}\right)}{\sum }S\left(R_{c1},R_{c2},...,R_{cn}\right)$$ (7)

H_*c*_ is the global representation of the clinical record, which summarizes the feature blocks of the clinical record. Then in the same way, we obtain the global representation of the time series data H_*t*_. To obtain multimodal contextual information, we compute the sum of the elements of the global representation for each modality, which generates the multimodal global representation K_*g*_:

$$K_{g}=elem\left(\sum \left(H_{c},H_{t}\right)\right)$$ (8)

The multimodal feature representation contains rich global contextual knowledge. Then, we apply a ReLU activation function on K_*g*_ to capture the dependencies between the multimodal features and map K_*g*_ to the joint representation Z, which helps the generalization of the model:

$$Z=w_{z}K_{g}+b_{z}$$ (9)

where w_*z*_ and b_*z*_ are the weights and biases. We generate the corresponding logits $U_{m}^{i}$ by linearly transforming Z and obtain the block-level attention weights $A_{m}^{i}$ by softmax activation. $W_{m}^{i}$ and $b_{m}^{i}$ are weights and bias of the corresponding fully connected layer.

$$U_{m}^{i}=W_{m}^{i}Z+b_{m}^{i}$$ (10)

$$A_{m}^{i}=\frac{exp\left(U_{m}^{i}\right)}{\overset{M}{\underset{k}{\sum }}\overset{\left|B_{k}\right|}{\underset{j}{\sum }}exp\left(U_{k}^{j}\right)}$$ (11)

The soft attention in the original MSAF depends on the total number of feature blocks, and the extracted features are suppressed. In particular, the suppression effect is more pronounced in complex tasks. By analogy with the medical field, there is a close correlation between the change process of patients’ health conditions and the clinical data generated during hospitalization, but soft attention suppresses this correlation and thus prevents accurate prediction. Therefore, we apply the soft attention mechanism at the modal data level to strengthen this correlation by weighting the average, while giving more weight to the more important parts of each block:

$$B_{m}^{i}=\left[\lambda +\left(1-\lambda \right)\times A_{m}^{i}\right]⊙\overset{i}{\underset{m}{B}}$$ (12)

$$F_{g}=\left[B_{m}^{1},B_{m}^{2},...,B_{m}^{\left|B_{m}\right|}\right]$$ (13)

*λ* ∈ (0,1) can be interpreted as a hyperparameter with control weights. We obtain an optimized feature block $B_{m}^{i}$ using attention signals $A_{m}^{i}$ and *λ*. Finally, the feature blocks belonging to modality m are merged by channel-wise concatenation to produce F_*g*_.

The article "Deep multi-modal intermediate fusion of clinical record and time series data in mortality prediction" was retracted in 2025. Reasons: plagiarism; overlap with other authors' work; concerns about the article.

Algorithm 1 The multimodal fusion model.

1: Initialize clinical record, time series data, and feature blocks of clinical records and time series R_*c*_, R_*t*_
2: **for** *i* = 1; *i* < *n*; *i* + + **do**
3: R_*c*_ = (R_*c*1_, R_*c*2_, …, R_*cn*_) # clinical record embedding
4: R_*t*_ = (R_*t*1_, R_*t*2_, …, R_*tn*_) # time series embedding
5: The multimodal fusion module associated with R_*c*_ and R_*t*_
6: The attention mechanisms learns to emphasize the important feature blocks
7: **end for**
8: Process the multimodal fusion matrix F_*g*_
9: Fusion state information, F_*g*_ and R_*t*_
10: Calculate the final risk score for death11: Perform prediction for test set and observe prediction performance

### 3.5 Mortality prediction

To be able to further capture the dependencies between modalities, we input the multimodal fusion representation F_*g*_ to the GRU layer to obtain the feature representation F_0*g*_. However, data offset may occur when data fusion is performed on different modal data. To compensate for this lost information and to represent patient information more comprehensively, the low-level feature representation extracted from the time series data is used for prediction along with the multimodal fusion features.

To fuse the multimodal features, we first connect the features *p* = concat (R_*t*_, F_0*g*_) to obtain a final multimodal fusion matrix for the patient. This matrix is then passed through a fully connected layer to predict the patient’s mortality using sigmoid as the activation function. Finally the predicted results are output.

## 4 Experiment

In this section, we conduct experiments on the real-world medical dataset MIMIC III to evaluate the performance of model. Compared with the baseline prediction model, the model achieves better results under different evaluation strategies.

### 4.1 Data description

#### 4.1.1 Dataset

We use a free and open, publicly available resource for intensive care unit research databases, MIMIC-III published on PhysioNet. The dataset includes 46,520 patients and contains identified comprehensive clinical monitoring device waveform data and rich clinical text records from the Intensive Care Unit (ICU) at Beth Israel Deaconess Medical Center between 2001 and 2012. The content of MIMIC-III includes vital signs, laboratory and radiology reports, treatment information, and more.

#### 4.1.2 Pre-processing

To prepare our in-hospital mortality dataset, we start with the root cohort and further exclude all ICU stays with unknown length of stay, length of stay less than 48 h, or no observed length of stay within 48 h. This yields a final training set and test set of 17,903 and 3,236 ICU stays, respectively. We determined in-hospital mortality by comparing the date of patient death with the time of admission and discharge. The resulting mortality rate was 13.23 (2,797 of 21,139 ICU stays). Because time-series data need to be combined with clinical records, clinical records collected within 48 h of the patient’s admission are required. After these steps, our dataset consisted of 11,579 records in the training set, 2,570 records in the validation set, and 2,573 records in the test set.

The article "Deep multi-modal intermediate fusion of clinical record and time series data in mortality prediction" was retracted in 2025. Reasons: plagiarism; overlap with other authors' work; concerns about the article.

For the time series part of the model, we first restricted the time series data to the first 48 h of the patient’s hospitalization, and then we resampled the time series data to a 1-h interval. We performed forward imputation on the missing values if they were generated. If no previous values were recorded, we used the pre-set values of the features given in Harutyunyan et al. (2019). After preprocessing the time series data, we used the LSTM network. We input the entire time series data of the patient into the LSTM model. For the clinical record part of the model, we use a fine-tuned BERT-based model for modeling clinical record, then we feed each clinical record of a patient separately to the text part of our model, and then combine the resulting embeddings to get the final representation of text part of the data.

### 4.2 Experiment setup

In this section, we first describe the state-of-the-art methods used for mortality prediction as a baseline, and then outline the metrics used for evaluation. Finally, we detail the implementation details. Baseline models. We compare our method with the baseline method for mortality prediction. The baseline model is as follows:

1) LSTM: Time series data processing with LSTM.
2) Bert: Clinical record processing with Bert.
3) CNN + LSTM: Clinical record processing with CNN, time series data processing with LSTM.
4) CNN + GRU: Clinical record processing with CNN, time series data processing with GRU.
5) Bert + LSTM: Clinical record processing with Bert, time series data processing with LSTM.
6) BioBert + LSTM: Clinical record processing with BioBert, time series data processing with LSTM.

These unimodal baseline models were selected for LSTM, and Bert processed the time series and text separately. These multi-modal baseline models are all combined for mortality prediction by replacing the unimodal data processing methods, and all use the commonly concat method for fusion and prediction before entering the fully connected layer.

#### 4.2.1 Evaluation strategies

Since in-hospital mortality prediction is a binary classification task with unbalanced categories (only about 10 of patients in this dataset suffered death), the area under subject working characteristics (AUC) was used to evaluate our model. We also report the area under the precision-recall curve (AUC-PR) metric because it can be more informative when dealing with highly skewed datasets.

#### 4.2.2 Implementation details

We implemented all baselines and models using pytorch. For the training model, we used Adam with a batch size of 5, an initial learning rate of 2e-5 for training, and a weight decay of 0.01. Training was terminated after 10 epochs because the evaluation value no longer improved as the number of epochs increased. We randomly divided the dataset into a training set, a test set, and a validation set in the ratio of 7:1.5:1.5.

The article "Deep multi-modal intermediate fusion of clinical record and time series data in mortality prediction" was retracted in 2025. Reasons: plagiarism; overlap with other authors' work; concerns about the article.

### 4.3 Performance evaluation

#### 4.3.1 Overall performance

Table 1 demonstrates the performance of the proposed model and the baseline of predicted mortality in the MIMIC-III dataset. The results show that the model outperforms all baselines. We note that in the real public dataset, the AUCPR of LSTM is lower than other models and the AUCROC values are slightly lower, mainly because LSTM uses a model with padding for missing values, so it does not capture the dependencies and correlations between different time series. CNN, Bert, BioBert and our model can capture the dependencies between medical texts and take into account all patient visits.

**TABLE 1:** Performance comparison on MIMIC-III data.

Model type	Model	AUCROC	AUCPR
Single-modal	LSTM	0.8333	0.4418
	GRU	0.8151	0.4931
	CNN	0.8374	0.4862
	Bert	0.8386	0.465
	BioBert	0.8553	0.5031
Multi-modal	CNN + LSTM	0.8486	0.5274
	CNN + GRU	0.8358	0.5136
	Bert + LSTM	0.8458	0.5215
	BioBert + LSTM	0.8724	0.5404
	BioBert + LSTM + Fusion	0.8835	0.5632

In the multi-modal fusion method, early fusion may contain a large number of redundant input vectors, while late fusion cannot capture the correlation between the underlying features of different modes. As can be seen from Table 1, compared with CNN + LSTM, CNN + LSTM and Bert + LSTM models that use concat to concatenate the data of the two modes before the decision, the middle fusion module we use makes the model perform better. Compared to the best-performing BioBert + LSTM, AUCROC improved by 1.1%, AUCPR improved by 2.28%. This is because the heterogeneity of multi-modal data makes the parameter space too complex to be determined by simple heterogeneous splicing. Our model can model different types of input and use different types of data to learn important characteristics, and the fusion module used can capture the correlation between different modes to help prediction. Compared with the simple splicing of multi-modal data for prediction (CNN + LSTM), our fusion method significantly improves the prediction performance of the model.

In order to prove the effectiveness of the performance improvement brought by multi-modal feature fusion, we also conducted experiments based on the original single-modal feature used by each model. It can be seen from Table 1 that the model performance is improved after the data of other modes are introduced. For example, in the BioBert + LSTM model, the ARUROC, AUCPR were improved by 2.8%, 3.7% respectively, after the clinical records were combined with the time-series data for prediction. This proves that information complementarity between multi-modal features can indeed enable models to better understand patient health and achieve higher predictive performance. This is also verified by the model based on GRU. The performance of the model proposed by us is significantly improved compared with that of GRU based on a single mode.

The article "Deep multi-modal intermediate fusion of clinical record and time series data in mortality prediction" was retracted in 2025. Reasons: plagiarism; overlap with other authors' work; concerns about the article.

### 4.3.2 Robustness for number of clinical-record

Tables 2–5 show the prediction results of mortality for four different numbers of clinical records. Compared with the baseline model, our proposed model performed best in terms of AUCROC, AUCPR performance indicators. The multimodal model always works better than the unimodal model in different numbers of clinical records.

**TABLE 2:** Performance of each model in the one clinical record.

Model	AUCROC	AUCPR
CNN + LSTM	0.8124	0.5026
CNN + GRU	0.8058	0.4847
Bert + LSTM	0.8186	0.5034
BioBert + LSTM	0.8327	0.5138
BioBert + LSTM + Fusion	0.8432	0.5256

**TABLE 3:** Performance of each model in the 4 clinical record.

Model	AUCROC	AUCPR
CNN + LSTM	0.8236	0.5095
CNN + GRU	0.8135	0.493
Bert + LSTM	0.8227	0.5089
BioBert + LSTM	0.8485	0.5214
BioBert + LSTM + Fusion	0.8637	0.5362

**TABLE 4:** Performance of each model in the 7 clinical record.

Model	AUCROC	AUCPR
CNN + LSTM	0.8367	0.5168
CNN + GRU	0.8287	0.5057
Bert + LSTM	0.8365	0.5136
BioBert + LSTM	0.8683	0.5367
BioBert + LSTM + Fusion	0.8752	0.5485

**TABLE 5:** Performance of each model in the 10 clinical record.

Model	AUCROC	AUCPR
CNN + LSTM	0.8486	0.5274
CNN + GRU	0.8358	0.5136
Bert + LSTM	0.8454	0.5215
BioBert + LSTM	0.8725	0.5404
BioBert + LSTM + Fusion	0.8835	0.5632

To assess the value of using multiple clinical records for each patient, we tried including a different number of clinical records for each patient in the different model. Figure 2 and Figure 3 shows the experimental results of the model when predicting different numbers of clinical records. It can be observed that the performance of the model in terms of both AUCROC and AUCPR rises as the number of clinical records increases, with the best performance being achieved when all clinical records are used.

**FIGURE 2:** Models’ robustness comparison of AUCROC.

**FIGURE 3:** Models’ robustness comparison of AUCPR.

### 4.3.3 Data ablation study

We conducted data ablation experiments based on the proposed model to examine the contribution of various data to the prediction task. First, as seen in Table 6, it is higher than a single model in all two evaluation metrics, suggesting that combining multiple models yields richer information about the patient and allows better monitoring of the patient’s condition. It is logical that the combination of different kinds of data can be complementary information. However, the predictive performance of the pure time series model is low because time series data have many missing values due to irregular sampling. This can have some impact on model learning. Clinical records are highly correlated with the patient’s physical condition, and models based on clinical records perform better than time series.

The article "Deep multi-modal intermediate fusion of clinical record and time series data in mortality prediction" was retracted in 2025. Reasons: plagiarism; overlap with other authors' work; concerns about the article.

**TABLE 6:** Data Ablation Results (T for time-series, C for clinical records).

Model	AUCROC	AUCPR
BioBert + LSTM + Fusion-T	0.8257	0.5048
BioBert + LSTM + Fusion-C	0.8465	0.5283
BioBert + LSTM + Fusion	0.8835	0.5632

## 5 Conclusion

Clinical records written by healthcare professionals include important information about the patient’s history and current status in the hospital, which can be used to significantly improve mortality prediction. In this work, this paper utilizes time series data and clinical records for mortality prediction to improve the monitoring of patients’ clinical health status. To overcome the drawbacks of unimodal data, We propose a multimodal fusion model that integrates multimodal data into the same architecture by improving the fusion module. Our proposed improved module partitions the features of each modal channel into feature blocks of equal size and then learns to emphasize the important feature blocks by generating attention values. Subsequently, the augmented feature blocks are reconnected for each modality to obtain an optimized feature space for understanding multimodal contexts. It captures the global information of a single modality and the relationship between multiple modalities, which helps to improve the predictive performance of the model. The performance of the model is validated on a real electronic medical record dataset, and the results show that our proposed model has good performance.

Semantic conflict repetition in current deep learning multimodal fusion models. The problems such as noise are still unresolved. Although attention mechanisms can solve part of the problem. But they work implicitly. Not actively controlled. Studying an active control can better combine logical reasoning and deep learning. How to solve the problem of unobstructed interoperability of information across modalities? How to solve the model generalization ability? These questions are the shortcomings of current multimodal models.

In the future, we want to solve the semantic conflict repetition, noise problem in deep learning multimodal fusion models.

The article "Deep multi-modal intermediate fusion of clinical record and time series data in mortality prediction" was retracted in 2025. Reasons: plagiarism; overlap with other authors' work; concerns about the article.

## Data Availability

The original contributions presented in the study are included in the article/Supplementary Material, further inquiries can be directed to the corresponding authors.
